# Application of sewage sludge combined with thiourea improves the growth and yield attributes of wheat (*Triticum aestivum* L.) genotypes under arsenic-contaminated soil

This article has been retracted.

**DOI:** 10.1371/journal.pone.0259289

**Published:** 2021-11-04

**Authors:** Nida Mansoora, Shameem Kausar, Syeda Fasiha Amjad, Samia Yaseen, Huma Shahid, Khadija tul Kubra, Saad A. M. Alamri, Sulaiman A. Alrumman, Ebrahem M. Eid, Ghulam Mustafa, Saleha Ahmed Ali, Subhan Danish

**Affiliations:** 1 Department of Botany, University of Agriculture Faisalabad, Punjab, Pakistan; 2 Department of Food Sciences, University of Agriculture Faisalabad, Punjab, Pakistan; 3 Biology Department, College of Science, King Khalid University, Abha, Saudi Arabia; 4 Botany Department, Faculty of Science, Kafrelsheikh University, Kafr El-Sheikh, Egypt; 5 Department of Soil Science, Faculty of Agricultural Sciences and Technology, Bahauddin Zakariya University, Multan, Pakistan; 6 Department of Botany, University of Lahore, Lahore, Punjab, Pakistan; Harran Üniversitesi: Harran Universitesi, TURKEY

## Abstract

Arsenic (As) contamination is a serious threat to agriculture and human health worldwide. It can adversely affect the growth attributes of food crops. On the other hand, using thiourea (TU) to ameliorate As stress is an economically consistent approach. However, there is a knowledge gap regarding the combined use of TU and Sewage sludge (SS). SS is considered important, unutilized biomass. It can be used as a fertilizer that has high organic matter and nutrients. Therefore, the current study was performed to evaluate TU and SS sole and combined responses under As toxicity on two wheat genotypes (Markaz 19 and Ujala 16). There were four treatments control (As 50 mg kg^-1^), SS (30 g kg^−1^)+TU (6.5 mM)+As, TU+As and SS+As applied with four replications. Results revealed that SS+TU performed significantly better over SS, TU and control for improvement in root and shoot fresh and dry weight of wheat varieties Markaz 19 and Ujala 16 under As toxicity. A significant decrease in POD, SOD and APX of Markaz 19 and Ujala 16 also validated the effective functioning of SS+TU over control. The maximum increase of 71 and 77% was noted in phosphorus, where SS+TU was applied over control in Markaz 19 and Ujala 16, respectively. In conclusion, SS+TU is a better approach than the sole application of SS and TU under As contamination for improvement in wheat growth attributes. More investigations are recommended at the field level under different As contamination and agro-climatic zones to declare SS+TU an effective amendment to mitigate As toxicity in wheat.

## 1. Introduction

Climate changes, environmental pollution, and ever-increasing population growth are major food safety concerns regarding human health [1]. Among abiotic stresses (i.e., drought, salinity, nutrition), heavy metals contamination deteriorate a large agricultural area [2–9]. Soil metal contamination is widespread worldwide in huge land areas, especially in Asian countries, including Pakistan [10–20]. Arsenic (As) is a toxic metalloid ubiquitously present in the soil at trace quantities normally [21]. Being a potential agricultural hazard, As contamination creates serious issues on a wide scale for sustainable crop production and food safety. Higher concentrations of arsenic in soil are phytotoxic in plants, decreasing plant growth and yields, stunted and discolored roots, yellow and withered leaves, less protein contents, and reduction in chlorophyll levels and photosynthetic capacity [10].

Furthermore, the transfer of As from growing media to cereal crops is a serious threat to human health. Its permissible limits worldwide are 5mg kg^−1^ and are increasing significantly in agricultural soils [4]. Industrial activities, i.e., coal combustion, glass manufacture, metal smelting and the use of pesticides, fertilizers and desiccants having arsenic contents, highly increased its levels [22].

Counteracting As stress, supplementation of non-physiological sulfur-containing TU can ameliorate metal stress in wheat plants via an antioxidant defense system and improvement of redox status. Also, TU is a cost-effective compound in comparison with other similar chemical compounds. Sulphur in TU is a constituent of tripeptide glutathione involved in detoxifying arsenic and ROS scavenging to keep the system optimal. The effect of TU even acts at transcriptional regulation levels. It is considering physiological roles, TU increase plant photosynthetic performance, green pigments, and leaf growth. Arsenic toxicity results in photosynthesis decline and plant growth due to extensive ROS accumulation in cells. Since TU is a well-known ROS scavenger, it can effectively scavenge ROS [22].

Sewage sludge (SS) is a semi-solid and inevitably discarded waste material produced by wastewater treatments. The quantity of domestic wastewater and SS production has risen due to population expansion and urbanization. Its disposal is one of the main environmental concerns these days as it leads to environmental pollution. SS contains both macro-and micro-nutrients essential for plant growth and development. It seems a valuable addition of organic matter to the lands under cultivation instead of its dumping and safe management concerning ecological perspectives. It lowers the cost of expensive mineral fertilizers. The residuals and remnants used as organic matter in SS in cultivated lands are eco-friendly and broadly practiced. Wheat growth parameters and biomass significantly increase with SS when added in low concentrations to decrease the risk of heavy metal toxicity under their phytotoxic levels [23, 24].

Wheat (*Triticum aestivum* L.) is one of the most important crops in the world. Due to increasing metal toxicity, its net production is badly affected [25]. Metal toxicity resulted in a noticeable reduction in annual wheat production worldwide. Among 30 wheat varieties being developed in Pakistan, Markaz 19 and Ujala 16 are new ones. Both varieties have their nutritional requirements [26]. Ujala 16 has 14.7% proteins contents and 40 g 1000 kernel weight, while Markaz 19 has 15% proteins contents, 78.7 kg/hl test weight, a medium-maturing wheat variety, and adapted to rain-fed areas. Wheat production is inhibited by various biotic and abiotic stresses, including metal stress [27]. Its quality directly affects human food security and people’s lives [22]. The physiological activities of wheat plants were changed under arsenic stress. Its potential effects on wheat reduce the dry weight of root, stem, spike, and yield. The roots are supposed to have a high concentration of arsenic than upper above-ground parts [24].

In the recent past, several researchers focused on either supplementation of SS or application of TU separately to mitigate the adverse effects of heavy metals. There is not enough information on their combined application that has merely been tested as a valuable amendment in arsenic-contaminated soils. This study is helpful to cover the knowledge gap of comparison between sole and combined application of TU and SS effects on wheat under As stress. Therefore, the premier objective of the present study was to evaluate the effectiveness of the combined application of SS and TU to improve the performance of wheat under arsenic stress. It is hypothesized that wheat plants with supplementation of SS and TU might perform better under As stress than untreated plants.

## 2. Materials and methods

### 2.1. Experiment site

We conducted a pot experiment research field of Old Botanical Garden, University of Agriculture, Faisalabad. Faisalabad is located at 31.4504° N, 73.1350° E at 610 ft above mean sea level in flat plains of northeast Punjab in a semi-arid temperature zone with very hot, humid summers and dry, cool winters.

### 2.2. Seeds sterilization

Seeds of two wheat genotypes (Markaz 19 and Ujala 16) were collected from Ayub Agriculture Research Institute, Faisalabad. Markaz 19 was tolerant, while Ujala 16 was moderately sensitive against metals toxicity. All seeds were surface sterilized for 1 min using 95% ethanol and 10 min with 70% sodium hypochlorite solution (NaOHCl). Later, seeds were treated five times with distilled water to be washed.

### 2.3. Soil characteristics, seed sowing and application of treatments

The soil used in this experiment was coarse-silty loam, mixed thoroughly and sieved. For soil analysis, a sample from this soil was taken. Some soil properties are presented as Sand 19%, Silt 52%, Clay 7.82% [28], pH 7.5 [29], EC 0.5 dS/m [30], organic matter 0.4% [31] and arsenic 1.84 mg/kg [32]. Thirty-two plastic pots (23 cm diameter × 28 cm height) were filled with 5 kg soil portions. The soil was supplemented with 6.5 mM of thiourea and 30 g kg^−1^ of SS. Arsenic stress was given at a concentration of 50 mg kg^−1^ of soil [33–35]. Arsenic solution (Na_3_AsO_4_.12H_2_O) was mixed with the soil thoroughly at the control and other treatment (50 mg As/kg soil). After this, the soil was air-dried and again passed through a 2 mm sieve and let it settle for a week. SS used as organic fertilizer was taken local domestic site and was 50% amended. The SS was surface applied on pot soil with only one application in a single trance after adding arsenic to the soil. After a month of applying the treatments, wheat was sown at 2 cm soil depth in early October. Ten seeds were sown in each pot, and one week after germination, only seven healthy seedlings were maintained by thinning. The wheat was irrigated with good quality irrigated water. All chemicals used in this experiment were of analytical grades.

### 2.4. Experimental design and nutrients application

The experimental design was completely randomized (CRD) with four replications from each treatment. The combined treatments were as: (1) Control (with no TU, SS and As (50 mg kg^−1^)); (2) SS+TU: SS (30 g kg^−1^)+TU (6.5 mM) +As; (3) TU+As; (4) SS+As. To fulfil macronutrients requirement nitrogen, phosphorus and potassium fertilizers were applied at the rate of 120, 90 and 60 kg ha^−1^.

### 2.5. Harvesting and data collection

Plants were harvested after 35 days of sowing and analyzed for their morphological, physio- biochemical parameters. Fresh samples of leaves were collected randomly from each pot. The plants were washed using distilled water. Fully functional and healthy leaf samples from each treatment were selected for various pigments and enzymatic content studies. Root and shoot length, fresh and dry weight, total chlorophyll, chlorophyll a and b contents, carotenoids, total soluble proteins, soluble sugars, proline, malondialdehyde (MDA), H_2_O_2_, electrolyte leakage and contents like superoxide dismutase (SOD), peroxidase (POD) and ascorbate peroxidase (APX) were analyzed. Analysis of ions like sodium (Na), potassium (K), calcium (Ca) and phosphorus (P) was also evaluated.

### 2.6. Physiological attributes

Length of shoot and roots was measured with the help of a measuring tape. Immediately after harvesting, the fresh weight was measured by using a digital weighing balance. The samples were stored at -30°C for further fresh analysis. Wheat plants from each treatment were oven dehydrated for three days at 65°C [36]. These dried samples were used to measure the dry weight of roots and shoot and for ion analysis.

### 2.7. Estimation of photosynthetic pigments, total soluble proteins and soluble sugars

Total chlorophyll contents of leaves were estimated by following the Lichtenthaler and Wellburn [6] method. Chlorophyll a, b and carotenoid contents were analyzed following standard Arnon protocol [7]. About 0.1 g of fresh leaf samples were homogenized in 95% acetone (8 mL) at 4°C for 24 hrs. in darkness. Sample absorbance at 646.6, 663.6, and 450 nm was observed using a spectrophotometer (UV-2550; Shimadzu, Kyoto, Japan). Soluble sugars were determined by Dubois et al. method [37] while proteins contents were estimated following Bradford protocol [38].

### 2.8. Oxidative stress indicators

MDA contents were evaluated by triturating 0.1 g of leaf samples in 1% polyethene pyrrole solution and 25 ml of chilled phosphate buffer (pH 7.8) of 50 mM concentration at 4°C. The homogenous mixture was then centrifuged at 10,000g for 15 min at a low temperature. After heating at 100°C for 20 min, the mixture was immediately cooled down using an ice bath. Absorbance was observed at wavelengths of 450, 532 and 600 nm. Peroxidation of lipids was described as 1 mol g^-1^ following the protocol by Heath and Packer [39].


MDA=6.45×(A532−A600)−0.56×A450

H_2_O_2_ contents of wheat plant samples were determined by mixing 3 mL of the extracted sample with 1 mL of 0.1% titanium sulphate prepared in 20% H_2_SO_4_ v/v, and then homogenate was centrifuged for 15 min at 6000g. The irradiation of samples was evaluated at 410 nm wavelength by using a spectrophotometer. H_2_O_2_contents were assessed by extinction coefficient of 0.28 mmol^-1^ cm^-1^ [40]. Electrolyte leakage was evaluated by Anjum et al [41] protocol while proline contents in leaves were determined by Bates et al. [42] protocol.

### 2.9. POD, APX and SOD assay

Peroxidase (POD) activity was analyzed by using the methods of Sakharov and Ardila [43] according to which reaction mixture was prepared by mixing 0.05 mL of enzyme extract with 2.75 mL of phosphate buffer (50 mM, pH 7.0), 0.1 mL of H_2_O_2_ (1%), and 0.1 mL guaiacol solution (4%). Absorbance was recorded at wavelength 470 nm. The unit enzyme activity was accounted as the amount of peroxidase enzyme present.

The ascorbate peroxidase (APX) enzyme activity was evaluated by following Nakano and Asada method [44]. Beauchamp and Fridovich method [45] was used to assess the superoxide dismutase activity (SOD).

### 2.10. Determination of Na, Ca, P and K concentration in leaves

Plants were washed twice with redistilled water for the nutrient analysis. Plant samples were kept in the oven for three days at 65°C to be dried. The samples were then digested in HNO_3_: HClO_4_ 7:3 V/V solution by wet digestion method until a clear sample was obtained [46]. The samples were filtered, followed by dilution in redistilled water, and raised to 50 mL.

Yoshida et al. [47] proposed Ca, Na and K ions determination method in plants. Ionic concentration was measured by atomic absorption spectrum flame photometer. Concentrations of unknown samples of respective elements were found by constructing standard curves using standard series.

To determine phosphate contents, 2N nitric acid (2 mL) was added to digested material (1 mL), and the solution was diluted with distilled water up to 8 ml. After this, 1 ml of solution was mixed with molybdate-vanadate reagent solution (1 mL), and volume was maintained at 10 ml using distilled water. Absorbance was taken at 420nm [48].

### 2.11. Statistical analysis

The data were evaluated based on two-way analysis of variance (ANOVA) and the difference in treatments was determined. The least significant difference test (**p** < 0.05) [49] was used to examine the mean comparison test between treatments. The graphical demonstration of data was carried out by Origin 2021 [50].

## 3. Results

### 3.1. Growth parameters

A significant effect of treatments was observed on fresh root weight (A), shoot fresh weight (B), root dry weight (C), shoot dry weight (D), root length (E) and shoot length (F) of wheat varieties Markaz 19 and Ujala 16 under arsenic stress (50 mg As kg^-1^ soil) (Fig 1). Results showed that SS+TU were significantly best from control for improving the fresh root weight in arsenic-contaminated soils in Markaz 19 and Ujala 16. Treatment TU also differed significantly for root fresh weight in Markaz 19 and Ujala 16 over control. However, SS was non-significant in Markaz 19 but significant in Ujala 16 to enhance root fresh weight over control. For shoot fresh weight, SS+TU and TU were statistically similar to each other but were significantly better over control in Markaz 19. For Ujala 16 root fresh weight, SS+TU was significantly best than control. Treatments TU and SS were equally effective but differed significantly compared to control for an increase in shoot fresh weight in Ujala 16. It was observed that all the treatments, i.e., TU, SS and SS+TU were significantly different for root and shoot dry weight compared to control. For root length and shoot length, SS+TU was significantly best than control. However, maximum significant enhancement in root fresh, dry weight, root length and shoot length was noted in SS+TU than control.

**Fig 1:** Impact of treatments on growth root fresh weight (A), shoot fresh weight (B), root dry weight (C), shoot dry weight (D), root length (E) and shoot length (F) of two wheat genotypes (Markaz 19 and Ujala 16) after 35 d of growth in pots. All values are the mean of 4 replicates. Error bars are showing ± standard error. Different letters on bars are significantly different at **p** < 0.05 according to LSD test. C: Control, SS+TU: sewage sludge+thiourea, TU: thiourea, SS: sewage sludge.

### 3.2. Chlorophyll contents

Effect of treatments was non-significant for chlorophyll a (A), chlorophyll b (B), total chlorophyll (C) but significant for carotenoids (D) of wheat varieties Markaz 19 and Ujala 16 cultivated in As toxicity (Fig 2). Compared to control, treatment SS caused a significant decrease in chlorophyll a and total chlorophyll in Markaz 19. Application of TU remained non-significant for chlorophyll a, but significantly decreased total chlorophyll than control in Markaz 19. For chlorophyll b, all treatments remained non-significant over control in Markaz 19 and Ujala 16. For carotenoids, sole application, i.e., SS and TU remained non-significant over control in Markaz 19 and Ujala 16. However, treatment SS+TU caused significant improvement in carotenoids compared to control in Markaz 19 and Ujala 16.

**Fig 2:** Effect of different treatments on chlorophyll a (A), chlorophyll b (B), total chlorophyll (C) and carotenoids (D) of two wheat genotypes (Markaz 19 and Ujala 16) after 35 d of growth in pots. All values are the mean of 4 replicates. Error bars are showing ± standard error. Different letters on bars are significantly different at **p** < 0.05 according to LSD test. C: Control, SS+TU: sewage sludge+thiourea, TU: thiourea, SS: sewage sludge.

### 3.3. SOD, POD, APx and soluble sugars

Results showed that SS+TU significantly decreased SOD in Markaz 19 and Ujala 16 over control. Application of TU in Markaz 19 and Ujala 16 also caused a significant reduction in SOD than control. However, no significant change was noted in Markaz 19 and Ujala 16 where SS was applied compared to control (Fig 3A). For POD, treatments SS, TU and SS+TU remained significantly effective for a decrease over control in Markaz 19 and Ujala 16 (Fig 3B). In the case APX, treatment SS+TU differed significantly from control for the decrease in Markaz 19 (Fig 3C). However, no significant change was noted in Markaz 19 and Ujala 16 in APX and soluble sugar where SS, TU and SS+TU were added than control (Fig 3D).

**Fig 3:** Influence of different treatments on SOD (A), POD (B), APx (C) and soluble sugar (D) contents of two wheat genotypes (Markaz 19 and Ujala 16) after 35 d of the growth period in pots. All values are the mean of 4 replicates. Error bars are showing ± standard error. Different letters on bars are significantly different at **p** < 0.05 according to LSD test. C: Control, SS+TU: sewage sludge+thiourea, TU: thiourea, SS: sewage sludge.

### 3.4. MDA, H_2_O_2_, EL and proline contents

A significant decrease in MDA (Fig 4A) and H_2_O_2_ (Fig 4B) was observed where SS, TU and SS+TU were applied in Markaz 19 and Ujala 16. No significant change was noted in MDA of Markaz 19 among SS, TU and SS+TU. However, SS+TU significantly decreased MDA than SS in Ujala 16. In Markaz 19, SS, TU and SS+TU significantly decreased electrolyte leakage (Fig 4C) and proline than control (Fig 4D). However, only SS+TU caused a significant reduction in electrolyte leakage over control in Ujala 16. No significant change in proline was noted among all the treatments in Ujala 16.

**Fig 4:** Impact of different treatments on MDA (A), H_2_O_2_ (B), EL (C) and proline contents (D) of two wheat genotypes (Markaz 19 and Ujala 16) after 35 d of the growth period in pots. All values are the mean of 4 replicates. Error bars are showing ± standard error. Different letters on bars are significantly different at **p** < 0.05 according to LSD test. C: Control, SS+TU: sewage sludge+thiourea, TU: thiourea, SS: sewage sludge.

### 3.5. Ionic contents

Results showed that SS+TU differed significantly for improvement in phosphorus of Markaz 19 and Ujala 16. Treatments SS and TU were non-significant for Markaz 19 and Ujala 16 phosphorus. The maximum increase of 71 and 77% was noted in phosphorus, where SS+TU was applied over control in Markaz 19 and Ujala 16, respectively. In potassium and calcium, TU and SS+TU differed significantly from control in Markaz 19, respectively. However, in Ujala 16, all the treatments remained statistically alike for potassium and calcium. Treatments TU and SS+TU caused a significant decrease than control in sodium of Markaz 19 and Ujala 16. However, in total soluble proteins SS+TU remained significantly best for enhancement over control in Markaz 19 and Ujala 16 (Table 1).

**Table 1:** Effect of different treatments on ionic contents like sodium, calcium, potassium, phosphorous and soluble proteins constituents of two wheat genotypes (Markaz 19 and Ujala 16) after 35 d of the growth period in pots.

Treatments	Variety	Phosphorus	Potassium	Calcium	Sodium	Total Soluble Protein
		(mg g-1)	(mg g-1)	(mg g-1)	(mg g-1)	(mg g-1 FW)
**Control**	Markaz-19	1.33±0.06c	5.50±1.19bc	3.25±0.32bc	19.00±1.68a-c	3.00±0.26b
**TU+SS**		2.28±0.14a	8.25±1.11ab	6.38±1.07a	11.50±2.06e	4.30±0.05a
**TU**		1.42±0.13bc	9.25±0.48a	5.53±0.78ab	12.50±1.94de	2.53±0.27bc
**SS**		1.16±0.51c	5.25±1.11c	5.38±1.60ab	18.00±1.73a-d	2.45±0.19bc
**Control**	Ujala-16	1.23±0.05c	3.00±0.41c	2.38±0.63c	22.25±2.50a	2.15±0.31c
**TU+SS**		2.18±0.19ab	4.48±0.34c	4.00±0.20a-c	16.00±2.35b-e	3.03±0.37b
**TU**		1.17±0.14c	4.25±1.61c	3.88±0.52bc	14.50±1.32c-e	2.53±0.23bc
**SS**		0.91±0.43c	4.38±1.07c	3.25±0.48bc	21.00±2.12ab	3.13±0.26b

All the values are the mean of 4 replicates ± standard deviation. Different letters on bars are significantly different at **p** < 0.05 according to LSD test. C: Control, SS+TU: sewage sludge+thiourea, TU: thiourea, SS: sewage sludge.

## 4. Discussion

The contribution of organic matter in the soil plays an important role in nutrient recycling and relates to soil fertility sustainability. SS is considered an important strategy, especially in arid and semi-arid countries, such as Pakistan, where the soil organic matter is low [51]. Wheat is one of the world’s major food crops, and its productivity is suppressed by various environmental stress factors like heavy metal toxicity. A considerable agricultural land area is affected by arsenic contamination globally. Thiourea is well known for ameliorating metal stress in wheat plants and is economically a better choice among compatible compounds [25].

According to Yadav and Srivastava [22], a decline in photosynthetic pigments by As toxicity resulted in stunted plant growth, reduced biomass and plants height. Application of TU positively affected growth parameters. Several other studies further support that TU maintains source-sink regulatory processes in plants by enhancing metabolite translocation from leaves to other parts and increasing photosynthetic efficiency and dry matter contents [22, 52]. This mechanical feature of TU could be the fact behind reduced As toxicity in plants supplemented with TU. SS potentially improved soil nutritional quality, water-holding capacity and aeration, plant height, leaf biomass, leaf area, number of tillers, and wheat yield [53].

Tamrabet et al. [54] indicated that SS ameliorative effects are mainly derived from a net release of nitrogen contents from the decomposing organic matter present in SS with high nitrogen contents and less C/N ratio. The sewage sludge acts as a seal that reduces moisture evaporation from soil because of its high concentration of organic matter. Our study follows their results. Increase in fresh weight, dry matter accumulation and longer roots in Markaz 19 were more than Ujala 16 plants. Generally, SS treatments up to 40 g kg^−1^ shown a significantly positive effect in growth parameters and biomass of wheat than control [25]. A similar effect of SS was noticed in the current study.

The chlorophyll concentration was considerably decreased in wheat when subjected to As stress. It could be the metal-induced inhibition of protochlorophyllide reductase activity, which ultimately perturbed chlorophyll synthesis [10]. Arsenic toxicity is linked with adverse effects on photosynthetic pigments and efficiency of plants. A reduced concentration in pigment contents (chlorophyll a and chlorophyll b) was observed in only arsenic-treated plants of both varieties of rice [22]. Our results claimed that photosynthetic pigments increase in the combined application of SS+TU was more effective for Markaz 19 than Ujala 16. Samara et al. [51] reported the same results in wheat plants grown in a pot experiment. SS has great potential for improving and supplementing soil quality and describes this increase in biomass and morphometric parameters of wheat [55].

SS is one of the most important waste products due to its large production and disposal management worldwide. Agronomic use of sewage sludge is widely considered one of the useful treatments for several reasons, i.e., incorporating organic matter, nitrogen and phosphorous to the soil by improving its microbial, physicochemical, enzymatic properties and fertility [56]. The current experiment validates these previous findings.

The enzymatic antioxidants decreased when supplemented with SS+TU combined treatment in both genotypes. SS+TU and TU helped plants accumulating more soluble sugars in cells. Markaz 19 had comparatively lower Na and high Ca, P and K concentrations than Ujala 16.

Latare et al. [57] reported the decrease in soil pH under SS amendments. The decline in soil pH was attributed to the production of organic acids by SS supplementation in wheat [58]. SS mineralizes organic nitrogen to the soil, producing protons by nitrification and sulfur-compounds mineralization by decreasing soil pH. Srivastava et al. [59] observed a significant decline in protein contents occur due to arsenic contamination. Reduced protein levels in arsenic-treated plants are attributed to arsenic toxicity arbitrated via consequent protolysis and ROS production. Application of TU alleviated arsenic stress to plants and helped restore the protein level with regard to control value [60]. Similar effects of arsenic were found in current study. SS+TU treatment was proved more efficient in accumulating more proteins.

As stress causes enhanced ROS production and a burst of oxidative stress in plants [61]. Such as, in the current investigation, As stress (50 mg/kg) elevated MDA and H_2_O_2_ levels in wheat, showing ROS causing peroxidation of membrane lipids; the ROS-mediated lipid peroxidation leading to membrane leakage [62]. Therefore, more EL was observed in As stressed wheat plants. This association of ROS with EL and MDA commonly occurs when plants are subjected to stress conditions. Yadav and Srivastava [22] reported that the reduction in photosynthetic performance of plants is also due to enhanced ROS production upon stress. Since thiourea is the most important ROS scavenger, ROS species and increased antioxidant contents in cells might be effectively scavenged by thiourea. The application of SS showed highly significant effects in increasing K and P contents in soil [25]. Our results validate these facts. Arsenic stress increased ROS production while SS and TU had an ameliorating effect in decreasing reactive oxygen species.

Awasthi et al. [60] said that antioxidants play an important role in regulating ROS levels. SOD acting as superoxide radicals cause dismutation of free radicals and converted to hydrogen peroxide to be managed in cells via several other antioxidants. SOD level increased significantly in response to arsenic stress is in confirmation to earlier works of Chauhan et al. [63] and Awasthi et al. [60]. Arsenic toxicity amelioration mediated by thiourea and the reduction in ROS load was evident due to a reduction in antioxidant activities in applied treatments [51]. Decrease in ROS production and thus the oxidative stress in wheat eventually results in lowered arsenic toxicity and induction of tolerance as described by Srivastava et al. [59]. Our results are also in justification of these mechanisms regarding the use of SS and TU to prevent heavy metal contamination and recycling of sewage residuals feasibly and sustainably.

## 5. Conclusions

In conclusion, the application of TU and SS is effective for remediation of As toxicity. However, the combined application of SS and TU (SS+TU) is significantly better than the sole application. SS+TU also has the potential to improve carotenoids contents, phosphorus and potassium uptake in wheat under As contamination. However, SS+TU can also be played an imperative role in decreasing POD, SOD and APX in wheat under As stress. Farmers can improve the growth attributes of wheat varieties, i.e., Markaz 19 and Ujala 16 under As toxicity, by applying SS+TU. More investigations is yet suggested at the field level under different agroclimatic conditions to validate the results using SS+TU as an effective amendment for the alleviation of As stress in wheat.
